The article "Analysis of English Cultural Teaching Model Based on Machine Learning" was published in 2022. Journal: Comput Intell Neurosci.

# Analysis of English Cultural Teaching Model Based on Machine Learning

**DOI:** 10.1155/2022/7126758

**Published:** 2022-05-14

**Authors:** Qianqian Yang

**Affiliations:** School of Foreign Languages and Cultures, Beijing Wuzi University, Beijing 101149, China

## Abstract

According to the world population, nearly five billion people use mobile phones in their daily lives, and this has increased by 20% in the last twelve months compared to the previous report. An average survey conducted by researchers to find the amount of data consumed in a month by every mobile phone in the world has finally resulted in 45 exabytes of data being collected from a single user within a month. In today's world, data consumption and data analytics are being considered as one of the most important necessities for e-commerce companies. With the help of such collected data from a person, it is possible to predict the future signature or activity of the person. If 45 terabytes of data can be stored for a single user, determining the average calculation and amount of data to be collected for five billion users appears to be much more difficult. More than the human working concept, it looks like it would be difficult for a traditional computer system to handle this amount of data. To study and understand a concept from machine learning and artificial intelligence requires quite a collection of data to predict according to a person's activity. This article explains the roles of faculty and students, as well as the requirements for academic evaluation. Even before the pandemic, most people did not have any idea about the online teaching model. It is only after the disability of conducting direct (offline) classes that people are forced to get into the online world of teaching. Nearly 60% of countries are trying to convert their education systems to such online models, which improve communication between students and teachers and also enable different schemes for students. Big data can be considered as one of the technological revolutions in information technology companies that became popular after the crisis of cloud computing. A support vector machine (SVM) is proposed for analyzing English culture teaching and is compared with the traditional fuzzy logic. The results show the proposed model achieves an accuracy of 98%, which is 5% higher than the existing algorithm.

## 1. Introduction

College English teaching models are becoming more and more rigorous, making it harder to foster students' broad language abilities that are necessary for coping with globalisation and economic integration [1]. The substance, shape, strategy, and design of training will go through essential and key changes accordingly. The mix of media innovation and unknown dialect training has for some time been an intriguing issue for study, and it is likewise an interesting issue in 21st century unknown dialect education under the pattern of the profound mix of current data innovation and innovation. In 2004, 2007, and 2020, the Ministry of Education of China gave “School English Course Requirements (Trial),” “School English Course Requirements,” and “School English Curriculum Requirements,” which plainly expressed the PC-based media [2]. The English showing mode is a recently planned English program to assist Chinese undergrads with arriving at the necessary level for the educational plan. As long as students are encouraged to use the computer to its full potential in speaking and listening tasks, they will be able to achieve greater levels of individuality in their academic performance [3]. Teachers may also use computers to successfully teach reading, writing, and translation in order to assist students in enhancing their overall language abilities.

With the advancement of information technology, multimedia teaching has emerged in educational settings, offering significant benefits in terms of efficiency [4]. A teaching resource library in community nursing multimedia teaching may successfully increase students' interest in learning and maximize teaching outcomes. Reading comprehension and vocabulary retention were improved by adding YouTube to reading courses [5]. The research found that people who had seen YouTube clips performed better than those who had not. Using data from a survey of high school students, the author explores ways to motivate pupils to study English in a multimedia setting by using effective strategies. This is an essential “input and interaction” process that guarantees that the learner's demands are taken into consideration and that meaningful learning results are achieved. The author examined the intelligent classroom and multimedia system-based music education concept. Because of the vividness and real-time nature of today's technology, multimedia technology makes full use of the power of music software to create, change, and produce electronic music. According to this, teachers need to rethink their position since every kid has the ability to design their own curriculum, no matter where they are, thanks to advances in technology. Students will also need to master multimedia skills for cooperation and communication in the classroom [6]. Teachers may tailor their instruction to the individual needs of their pupils using multimedia-assisted language learning methods. Students may actively search for, ask questions, and answer questions about the information they are interested in or do not understand throughout the learning process. Instead of asking all pupils to work on the same assignment at the same time, computers provide each one with a personal instructor. For students with varying levels of language proficiency, specialization, and understanding ability, it is of particular benefit [7]. This means that although it may only take student A three days to complete the content that he is required to study in class, it may take the teacher up to an entire week for him to do so. By clicking the mouse frequently, if student B has challenges during learning, the issue and its resolution may be resolved and reinforced.

As a result of the Internet of Things allowing teachers to offer online software and exercises, many courses were previously unavailable via traditional means [8]. Students may choose the best English learning tools based on their personal conditions and development. Educators are often involved in the process of selecting educational resources [9]. Textbooks will become more student-centered as the class grows in size and diversity, allowing students more time to connect with their professors while making up for the time they would have spent in class if they all had the same abilities and skills. The most important factor is that users are not constrained by time or location in their selection of resources to be played [10]. Multiuser support, simultaneous transmission and presentation of resources, and the high quality of the resources are only a few of the benefits of using this method. It is possible to meet the demands of users with varying network bandwidths, offer users control features for replicating resources, and simultaneously analyze average resource flow statistics [11].

Students at a college or university may use multimedia education in a broad range of digital building projects on their campuses. Streaming media can be used to broadcast lecture materials to students all over the world via a network, allowing professors to focus on other aspects of their classes while their students can learn from anywhere [12]. Streaming media technology may help students learn more effectively in the self-study industry since many online resources create a stimulating learning environment, yet text-based materials are often boring. It is very uncommon for notable professors and specialists to give lectures on campus, and these lectures are streamed live online [13]. Overcrowding is a common problem when there is a large number of attendees. It is possible to broadcast on-site situations in real-time using multimedia teaching technology, allowing for the real-time dissemination of lectures to students. It is possible to make on-demand watching of entertainment materials possible via audio university's multimedia education. As a university, it is possible to turn cultural events, sporting events, and other activities that take place on campus into resources and deploy them on the server so students may access them [14].

English is one of the most commonly spoken languages in the world and one of the most important languages in the international community. Today, the trend of globalization is speeding up significantly [15]. English is an essential language for pupils who want to travel throughout the globe. In addition to expanding their horizons and enhancing their personal benefits, learning English may boost their knowledge. Composition writing in English is a need for everyone studying the language. In addition to fundamental information such as vocabulary and grammar, writing may also represent students' general comprehension of sentence structure, discourse, and logical reasoning abilities [16]. The ability to write in English is a clear indicator of a student's overall proficiency in the language. Hence, test organizers focus on this skill when assessing students' language proficiency. This has resulted in a growing number of students paying attention to it. Teaching staff must spend a lot of time on writing since it is a weak link in students' English learning at the moment [17]. When instructors assess them by hand in the normal learning environment, it is appropriate for a modest number of short English works. As essay length and marking requirements increase, this system will become less effective and more prone to mistaken conclusions [18]. Furthermore, manual grading is very subjective, and people from different backgrounds and places might have very different opinions about the same piece of writing.

There has been a tremendous increase in the use of Automated Essay Scoring (AES) technology in education because of the fast advancement of computer technology in recent years [19]. Although it can intelligently assess and grade writing, this technology has its limitations. Computer evaluations are less expensive and more efficient than human evaluations. To the degree that computers are adept at repetitive labor, the automated scoring system allows instructors to free up their physical and mental power, allowing them to dedicate more time and energy to teaching and research [20]. While students may use the findings of the analysis to improve their own writing via systematic recommendations for the correction of spelling and grammar issues, the other option is to use the data to offer feedback on further assessment information. The analysis findings might also offer fantastic phrases and sentences and composition elements to help students with their scientific writing. This paper's content statistics are being used to build and evaluate AES systems at this time. This inquiry does not go into great depths or with great accuracy, but it is simple enough to get a general idea [21]. As a consequence, while improving the predicted score accuracy, people also need to extensively study the composition's substance to ensure that the AES method can be correctly applied to actual composition correction.

There are numerous domains of multidisciplinary study that are involved in machine learning, and it is commonly employed in intelligent systems. Automated learning is the process through which a computer or machine learns from its complete experience and uses that knowledge to enhance its performance going forward. The future of work and the workforce will be profoundly affected by advances in machine learning [22]. The demand for machine learning products and the work tasks, platforms, and specialists required to develop them has risen as a result of the increasing usage of machine learning in a wide variety of industries. Using computers to do complicated analysis, nuanced judgment, and innovative problem solving, machine learning has a significant economic influence. Knowledge-based labor automation is being fueled by the development of deep learning and neural network machine learning. Also, driving machine learning technology are natural user interfaces for voice and gesture recognition. There has been a lot of interest in machine learning across a variety of sectors. Multiple classifiers may be dealt with using the Bayesian technique, *K*-means, or a neural network [23]. Powerful neural networks can handle nonlinear multiple classifiers with ease. For high-dimensional parameters, neural networks have a more sophisticated hidden layer than other approaches. In addition to this, the study evaluated the teaching and learning management of the English course with the student's behavior towards the online English course. The results show that the student's response to the classes is increased with the involvement of artificial intelligence technology with the Internet [24]. This study focused on analyzing an English cultural teaching model based on machine learning.

## 2. Materials and Methods

Until the growth of big data algorithms, the education system in China was not very popular and considered one of the notable things. After analyzing its benefits and new requirements, it creates a stable and sustainable education for students. If a teacher wants to teach a concept to a student, before that, they should get trained on the concept and also know how to relate such a concept with real-time applications to make it clear while teaching. Self-update is also an important way to improve the students' knowledge. If the teacher fails to update themselves with the current technological growth, then the faculty trained students will be affected once they get into the IT field. To solve the problem and to reduce the teacher's involvement, the systems are designed to analyze the market and update the students' learning syllabus accordingly. Here, the data collection is kept and stored in a cloud computing method to access its future purpose. According to the security guidelines, if the cloud-stored systems are kept private, then they can be used by any person at any time, even if the users are from different countries. In view of different learning methods (online and offline), the purpose of big data is being used more for the development of students' knowledge than what they get from offline classes (Figure 1). In this figure, artificial intelligence (AI) technology is implemented to automate the system process in the teaching mechanism. Machine learning (ML) technology is utilized for statistical analysis of the effective teaching process and to iterate the process with improved methodologies. Deep learning (DL) plays a vital role in filtering information. In this application of the English cultural teaching process, this DL mechanism will aid in the filtering of the students based on their level of learning to improve their learning process.

To form a well-developed education system, language is considered as the pillar for the delivery of such content to the students. Authors like Gardner and Lambert believe that there are two different types of motivation behind the research background of big data, which are instrumental motivation and “integrated” motivation. Both types are used to show the actual target language culture. Normally, to increase the learning platform, students' involvement and their interest are two of the most important things, and they can be separated into two different prospects, for example, internal motivation and external motivation. At the same time, internal and external motivation can be said to be the same when students are forced by external influences to get into the course. While gathering such data that is stored in the differences in the learning motivation, it can be divided into three different regions. One is about the value component, the second shows the expectation component, and the final thing deals with the emotional component. Students used to come from different fields, for example, lower education, higher education, undergraduate, Master's degree, and finally doctorate. Real time online and offline education on the English language and also cultural education through English have been examined. It also includes the teaching of English cultural learning from different parts of the country.

According to the statistical report, the values are separated with two different opinions, which are the average value and the standard deviation. Finally, all three levels will not be significant in any case but the levels would rise according to the value component and the expected value would be 4 to 5 intermediate levels. After the collaboration of such things, it creates a situation where machine learning and deep learning are used with the help of big data.

The multiple processors machine English cultural teaching model algorithm would be incorporated into a support vector machine (SVM), and the |*U*^*R*^(*τ*)*d*|^2^*ab*(*τ*) classification method of system modules would be launched within the SVM structure. Specifically, we will explain the English cultural teaching model creation approach and the ∑_*r*=0_^*R*^*∂*_2_*d*^2^,  ∀_*r*0_ ≥ 0 accompanying optimization technique based on a semisupervised multiprocessor English cultural teaching model. The following equation represents this teaching model:

(1) $$\begin{array}{c} \partial_{1}{\mathrm{||}d\mathrm{||}}^{2}\leq \int_{r_{0}}^{r_{0}+R_{0}}{\left|U^{R}\left(\tau \right)d\right|}^{2}ab\left(\tau \right)\leq \overset{R}{\underset{r=0}{\sum }}\partial_{2}{\mathrm{||}d\mathrm{||}}^{2},\;\forall_{r0}\geq 0. \end{array}$$

The sophistication of computation grows considerably as the structures  *∂*_1_*d*^2^ grow throughout this likelihood computation approach. The parameters of the model |*U*^*R*^(*τ*)*d*|^2^*ab*(*τ*) ≤ *∂*_2_*d*^2^,  ∀_*r*0_ ≥ 0 are practically impossible to gauge on present hardware. The presence of *f*^*p*^(*r*) in such a phrase is exclusively decided by the item preceding it. The framework for English cultural teaching is based on the following equation:

(2) $$\begin{array}{c} f^{p}\left(r\right)=\underset{g⟶0}{\lim}\frac{1}{g^{p}}\sum_{q=0}^{p}{\left(-1\right)}^{q}\left(\begin{array}{c} p\\ q \end{array}\right)f\left(r-qg\right). \end{array}$$

A sentence's similarity is measured exclusively by (∇^*a*^*x*/|∇^*a*^*x*|+*t*) , the two or more words before it. The framework for English cultural teaching is based on the following equation (the English cultural teaching model):

(3) $$\begin{array}{c} -\text{sent}\left(\frac{\nabla^{a}x}{\left|\nabla^{a}x\right|+t}\right)+\lambda_{e}\left(x-x^{0}\right)=0. \end{array}$$

The difference between the lim_*g*⟶0_ 1/*g*^*p*^ learner's cognitive level and the degree of difficulty to English cultural teaching model materials is indicated ∑_*q*=0_^*p*^(−1)^*q*^ by equation (4), where *q*_*i*_(*h*) is the student's language level target. Equations (3) and (4) specify the difference in cognitive level and the degree of difficulty in English cultural education through different models and materials is noted.

(4) $$\begin{array}{c} q_{i}\left(h\right)=\frac{f_{i}r_{i}-x\left(h\right)}{\lambda_{e}\left(x-x^{0}\right)}+\underset{g⟶0}{\text{lim}}\frac{1}{g^{p}}\sum_{q=0}^{p}{\left(-1\right)}^{q}. \end{array}$$

The learner's progress is indicated by *E*_*i*_^*n*^(*r*) the distinction between the learner's progress that helps the audience in grasping resource and knowledge sharing through English cultural teaching model where the learner wishes to gain information is represented in equation (5). The smaller the difference, the more closely the English Cultural Teaching Model resource's expertise points match *E*_*ij*_^*n*^(*r*) the learner's knowledge points.

(5) $$\begin{array}{c} E_{i}^{n}\left(r\right)=\underset{j\in L}{\sum }E_{ij}^{n}\left(r\right). \end{array}$$

(*u*, *w*; *A*, *ϕ*) the optimization technique of spending with both teaching programs represents the overall spending data using equation (6). English cultural teaching model material utilization is calculated.

(6) $$\begin{array}{c} \left(u,w;A,\phi \right)={\left|d\right|}^{-0.6}\int_{-\infty }^{+\infty }d\left(\tau \right)h\left(\tau -r\right)e^{-jb\tau }\text{d}\tau . \end{array}$$

The major purpose of the English cultural teaching model period *L*_*pp*_(*u*) objectives emphasize the disparities between the times required to complete the educational materials  *b*_*i*_*U*_*i*_(*u*)=*B*^*R*^*U*(*u*) and also the time designed to find the English cultural teaching model to determine the following equation:

(7) $$\begin{array}{c} L_{pp}\left(u\right)=\sum_{i=1}^{P}b_{i}U_{i}\left(u\right)=B^{R}U\left(u\right). \end{array}$$

The learner's total optimization performance, and  *ϕ*_*q*,*p*_ the English cultural teaching model route formed by the comments page function via recalculating coefficients, even though expressed by equation (8), is a functional illustration of the personalized English cultural teaching model route optimization method.

(8) $$\begin{array}{c} \phi_{q,p}=\frac{{\mathrm{||}Q\mathrm{||}}_{q,p}{}^{2}}{\delta^{2}}\text{exps}\left(\frac{\left(Q_{q,p}*A\right)}{3\delta^{2}}\right)*\left[e^{i\left(Q_{q,p}*A\right)}-e^{-\frac{\delta^{2}}{3}}\right]. \end{array}$$

The algorithm also *φ* classifies the notice of a particle propagation direction into three categories: speed resistance, self-English cultural education model, and social behavior. The ∑_*i*=1_^*O*^*Q*_*i*_*P*_*i*_/*U*(*Q*_*i*_ ∈ *Q*) stance update of material within generation has already been determined by a subatomic particle stance *t* formation and also the generation's motion direction, as explained below:

(9) $$\begin{array}{c} e=\frac{{\left(\varphi \phi_{35}+\varphi \phi_{04}\right)}^{2}+4\varphi \phi_{22}^{2}}{{\left(\varphi \phi_{35}+\varphi \phi_{04}\right)}^{2}}, \end{array}$$

(10) $$\begin{array}{c} B=\frac{\sum_{i=1}^{O}Q_{i}P}{\sum_{i=1}^{O}P_{i}}=\frac{\sum_{i=1}^{O}Q_{i}P_{i}}{U}\left(Q_{i}\in Q\right). \end{array}$$

From the standpoint of *Q*^″^ possibility, the state of *∂K*/*∂u*  particle has been defined. Each particle's *q*^″^ bit value within subspace is 0 or 1, and this particle calculation is just as described in the following equations:

(11) $$\begin{array}{c} Q^{\prime \prime }=\left\{Q^{\prime \prime }|q^{\prime \prime }=\frac{q^{\prime }\times n}{N},\;\forall q^{\prime }\in Q^{\prime }\right\}. \end{array}$$

(12) $$\begin{array}{c} \frac{\partial K}{\partial u}=\overset{p}{\underset{i=1}{\sum }}\left[h_{i}-\frac{\text{exps}\left(u+\sum_{j=1}^{q}u_{ij}\beta_{j}\right)}{1+\text{exps}\left(u+\sum_{j=1}^{m}u_{ij}\beta_{j}\right)}\right]=0, \end{array}$$

where *P*_*j* _ denotes the final method value of *j*, the amount of a existing final examination, and also the distinction here between the feature limitation levels of the *j* quantity. The differential factor's intensity is indicated by  *d*_*j*_. Because only the difficulty factor is considered, the optimization error can be mitigated to determine the following equation:

(13) $$\begin{array}{c} P=\sum_{j=1}^{4}P_{j}d_{j}+P=P_{4}d_{4}, \end{array}$$

where *P*_4_=|∑_*i*=1_^9^*s*_*i*3_*s*_*i*4_/∑_*i*=1_^9^*s*_13_ − ND| the final error between the ordinary problem of attempting to create exam papers and also the primary difficulty constraint of a defined test. The letter ND denotes a fictional test difficulty restriction. The distinction element of the major issues coefficient is denoted by *d*_4 _. Typically, this fitness is designed to be inversely proportional to the optimization process. The genetic algorithm can indeed be designed as follows to keep that common factor from being zero to determine the following equation:

(14) $$\begin{array}{c} R_{j}=\frac{1}{\left(1+\sum_{j=1}^{4}P_{j}d_{j}\right)}. \end{array}$$

It is obvious that the greater the F value, the better the quality of such a 1 scientific test. When *F* = 0, the best alternative that fits all of the constraints is found. Similarly, just this type of difficulty relationship can be simplified to the following equation:

(15) $$\begin{array}{c} R_{4}=\sum_{P⟶0}^{d}\left(1+P_{4}d_{4}\right)+E\sum_{d=1}^{t}1-d=1-\frac{e}{t}. \end{array}$$

The assessment difficulty is divided into four categories: challenging difficulties (*d* 〈0.4), more difficult situations (*d* 〈0.7), medium talks (0.4 ≤*d* ≤  0.7), and easy responses (0.6 ≤*d* ≤  1). The typical test paper challenge is organized as in the following equation:

(16) $$\begin{array}{c} \text{ND}=\frac{\sum_{i=1}^{n}\sum_{i=1}^{n}E_{i}k_{i}}{\sum_{i=1}^{n}E_{i}}. \end{array}$$

While ND means the ordinary difficulties of a test paper, *m* denotes the sequence of questions on the test paper, and *i* denotes the number of test questions, *i* = 0,  1,…*n*;  *E*_*i*_ signifies the difficulty of a *i* test, while *d*_*i*_ denotes the *i* test score. In this research, a wide range of analytical approaches is employed to determine the overall evaluation area score rate. To determine the score rate, the following equation is utilized.

(17) $$\begin{array}{c} D=\sum_{R⟶0}^{g}\frac{R_{T}-R_{O}}{g}+E_{g}\left(w\right)=\sum_{E⟶0}^{g}\left(\frac{g}{w}\right)E^{w}f^{g-w}. \end{array}$$

Every unbiased test results in the same probable outcome occurring but not occurring. Hence, this series of tests is known as just a heavy Binomial laboratory activity.

## 3. Result and Discussion

The |*U*^*R*^(*τ*)*d*|^2^*ab*(*τ*) system modules classification technique would be performed within the SVM framework. In particular, we will describe the English cultural teaching model creation approach, and also the accompanying optimization technique ∑_*r*=0_^*R*^*∂*_2_*d*^2^,  ∀_*r*0_ ≥ 0 based on a semisupervised nonlinear and non-English cultural teaching model. Based on the English cultural Teaching system in Figure 2, students must utilize machine learning approaches to scientifically establish the criteria, models, and processes required in the learning process in order to limit the likelihood of these issues.

People's goal is to create a novice educational environment within informatics courses through the use of novel instructional approaches known as a classroom setting. He also developed an artificial learning monitoring approach to help with the delivery of this course. The innovative group employs inverted teaching education, whereas the control group employs classroom instruction.

Based on the foregoing analysis, woman's performance is examined, and English online teaching is integrated to suitably qualify for learning behavior. The classification of 30 students in English online/offline learning is investigated, and also the teaching efficiency of 30 respondents is evaluated.  Table 1 displays data on student wearable sensors.

In Figures 2, and 3, *x* axis represents the number of classes for an online course that specifies to create a novice educational environment within informatics courses through the use of novel instructional approaches known as classroom settings. He also developed an artificial learning monitoring approach to help with the delivery of this course. The innovative group employs inverted teaching education, whereas the control group employs classroom instruction. Hence we specify for the natural numbers. The difference between the learners cognitive level lim_*g*⟶0_ 1/*g*^*p*^ and the degree of difficulty to English cultural teaching model materials ∑_*q*=0_^*p*^(−1)^*q*^ is indicated by equation (4). *q*_*i*_(*h*) represents the student's language level which is the target based in determining the learning level, and the analysis results are given in Figure 3; regression monitored and unsupervised learning are used as the research platform for building an English online teaching evaluation method, with a focus on problems such as semisupervised multilabel learning. These problems are common in the field of artificial intelligence, and there has been a lot of research done on them. Unlike previous studies, this paper employs matrix completion and generative structures to reinterpret such two problems in a different light and test the effectiveness of multiple simulation studies and actual data sets.

The investigation is carried out primarily through the use of the following methods: evaluation but also systematic evaluation. It is assumed that professional evaluation will be used in its assessment. The following methods are commonly used for checking: evaluation and organized evaluation. It is also assumed that evaluation employs evaluation methods because the artificial evaluation process is used to assess the testing process' accuracy.  Table 2 displays the assessment results of this document, which examines the students' merits of 20 teachers.

The English cultural teaching model period *L*_*pp*_(*u*) objectives emphasize the disparities between the times required to complete the educational materials  *b*_*i*_*U*_*i*_(*u*)=*B*^*R*^*U*(*u*) is the time designed to find to level of understanding in online teaching, and the results are illustrated in Figure 4 the framework developed in this paper is similar to the results of the manual analysis with an inaccuracy of no more than 4%. Because the manual ability to score performance in this document is fairly accurate, the system's ability to score performance is also accurate and reliable. As the result shown in Table 3, it can be concluded that the system developed in this paper has a positive effect just on teaching evaluation and it can be implemented to teaching and learning. Student Behaviour recognition is recorded to identify the effective result of English cultural education through online mode.

The methodology also  *φ* categorizes particle propagation direction notice into three categories: speed opposition, self-English cultural education framework, and social behavior. Subatomic stance *t* formations and the generation's movement direction have already determined the ∑_*i*=1_^*O*^*Q*_*i*_*P*_*i*_/*U*(*Q*_*i*_ ∈ *Q*) stance refresh of a substance within the generation. In Figure 5 based on the results of the preceding analysis, it is clear that the model developed in this paper has a positive impact on the recognition of students' actions and behaviors. Following that, this article considers teaching behavior. The evaluation is conducted primarily using two methods: analysis and thorough evaluation. Because it is assumed that evaluation employs expert assessment methods, the artificial evaluation process is used as a standard to assess the accuracy of a performance assessment.

Table 4 depicts the ratio result of the teacher education structure to evaluate the efficacy of the classroom learning framework to guarantee that there are no significant differences in all elements, excluding the various teaching methods. In this experimental study, the interactive behavior of the teaching strategy with students accounted for 60% of the total, which was higher than the proportion of interactive behavior with educators as the main structure (47.3%); the interactive behavior of the controlled group with students as the main structure accounted for 41.8%, which was lower than the quantity of interactive behavior with teachers (47.3%) (58% of the total).

It appears that the usage of SVM algorithms in the process of determining the optimum solution is significantly less than that of the random algorithm. Given the global lookup in SVM algorithms, the search variation is broad. People choose iterated ML material based on the best solution and search for the best solution's path, making it easier to identify the best solution. People could, in fact, build dynamic alteration parameters based on the results of the remainder of the experiment to effectively tackle the issue of inter objective, that is, a technique that provides test question document generation. When compared to the Fuzzy Clustering method, people were able to swiftly discover the ideal solution from the proposed algorithm. It provides for the best result in our proposed methods in SVM and is represented in Table 5 and Figure 6.

## 4. Conclusion

Nearly five billion individuals throughout the world use mobile phones on a daily basis, a 20 percent rise from the prior study during the last year. It took researchers an average of 45 months to gather 45 exabytes of data from users around the world in order to find out how much data each phone uses on a monthly basis. In today's environment, e-commerce enterprises must regard data consumption and data analytics as one of their most critical requirements. It is possible to forecast a person's future signature or activity with the use of such collected data. An average calculation and data collection amount for five billion users appear more complex when the data storage capacity for one user exceeds 45 terabytes. Before the pandemic, most people had no concept about Internet teaching. Direct (offline) classes cannot be taught any longer. Hence educators are forced into the online/offline classroom. 60% of countries are implementing online education methods that facilitate better contact between students and teachers and allow for a variety of student options. After the cloud computing disaster, a new wave of innovation called “big data” began to gain traction in the IT industry. The classic Fuzzy Logic is contrasted to a Support Vector Machine (SVM) for analyzing English Culture Teaching. The proposed model has obtained an accuracy of 98%, which is 5% greater than the current approach, according to the data.

## Figures and Tables

**Figure 1:** Big data collection for student monitoring system.

**Figure 2:** English cultural Teaching system design representation.

**Figure 3:** English cultural teaching model based on machine learning.

**Figure 4:** Statistical evaluation of the English cultural teaching model in behaviour recognition.

**Figure 5:** The recognition of Student and Teacher actions and behaviors for English cultural teaching model.

**Figure 6:** Performance of Comparison Result Analysis of two types of test papers.

**Table 1:** Descriptive statistical table of behavior patterns classification model for English online/offline teaching students.

No	Rate of action recognition (%)	No	Rate of action recognition (%)
1	92.77	16	94.34
2	94.89	17	96.29
3	95.80	18	95.65
4	86.43	19	92.94
5	92.34	20	92.45
6	97.53	21	85.69
7	95.24	22	96.38
8	98.95	23	92.27
9	97.57	24	94.63
10	92.78	25	94.12
11	94.74	26	95.81
12	96.12	27	97.20
13	95.67	28	91.47
14	93.38	29	96.27
15	86.78	30	98.92

**Table 2:** The result analysis of an evaluation of ML using English cultural teaching model.

No	Learning management	Teaching management
1	73.7	75.7
2	96.2	83.4
3	61.5	87.6
4	86.3	92.4
5	72.8	85.7
6	75.9	82.6
7	87.8	76.3
8	85.7	91.5
9	81.6	77.8
10	61.4	83.2
11	87.3	97.4
12	85.5	74.6
13	86.6	82.7
14	73.6	87.5
15	75.4	95.8
16	83.4	94.5
17	75.6	87.4
18	76.6	88.6
19	83.4	98.8
20	87.5	89.4

**Table 3:** Result statistical evaluation of the English online teaching behavior recognition.

No	English online teaching	Student behaviour recognition
1	91.77	95.34
2	95.89	98.29
3	93.8	93.65
4	89.43	91.94
5	91.34	90.45
6	93.53	89.69
7	97.24	97.38
8	95.95	95.27
9	96.57	94.63
10	91.78	96.12
11	92.74	93.81
12	97.12	94.2
13	98.67	92.47
14	94.38	97.27
15	89.78	95.92

**Table 4:** Result analysis for recognition of Student and Teacher actions and behaviors.

Recognition of student and teacher actions and behaviors using ML		
	Test group	Control group
Silence and chaos	2.8	1.7
Teacher interaction	47.3	58.4
Student interaction	51.9	41.8

**Table 5:** Algorithm comparison of two types of test papers.

Data set	Experimental number	Fuzzy clustering method (%)	Support vector machine (SVM) using ML (%)
Student performance data set	1	88	97
	2	93	99
	3	96	98

Overall accuracy (%)		93.66	98

## Data Availability

The data used to support the ﬁndings of this study are available from the author upon request.

## References

[1] Li P., Li C. (2017). Construction of multimedia teaching platform for community nursing based on teaching resource library technology. *International Journal of Emerging Technologies in Learning*.

[2] Kabooha R., Elyas T. (2018). The effects of YouTube in multimedia instruction for vocabulary learning: perceptions of EFL students and teachers. *English Language Teaching*.

[3] Philominraj A., Jeyabalan D., Vidal-Silva C. (2017). Visual learning: a learner centered approach to enhance English language teaching. *English Language Teaching*.

[4] Jin C. (2017). Analysis of music teaching mode innovation based on intelligent classroom and multimedia system. *Revista de la Facultad de Ingenieria*.

[5] Mpemba T. (2018). Reluctance to sanction Kiswahili instructional medium in post-primary education: how do the learners and their instructors cope with or resist the English medium policy?. *Phi delta Kappan*.

[6] Muslem A., Abbas M. (2017). The effectiveness of immersive multimedia learning with peer support on English speaking and reading aloud. *International Journal of Instruction*.

[7] Hennessy D. A. (2017). Conceptual models underlying economic analysis of animal health and welfare with the inclusion of three components: people, products and resources. *Revue Scientifique et Technique de l’OIE*.

[8] Carne C., Semple S., MacLarnon A., Majolo B., Maréchal L. (2017). Implications of tourist-macaque interactions for disease transmission. *Eco Health*.

[9] Farine D. (2017). The dynamics of transmission and the dynamics of networks. *Journal of Animal Ecology*.

[10] Santos L. M. D. A., Kadri M. S. E., Gamero R., Gimenez T. (2018). Teaching English as an additional language for social participation: digital technology in an immersion programme. *Revista Brasileira de Linguística Aplicada*.

[11] Zhang T., Luo Y., Sun Y., Li T., Qiu H.-J. (2018). New-concept animal vaccines emerging in recent years. *Sheng wu gong cheng xue bao = Chinese journal of biotechnology*.

[12] Kaldrymidou E., Kanakoudis G., Katsaras K., Tsangaris T., Papaioannou N. (2018). Bovine spongiform encephalopathy and public health. *Journal of the Hellenic Veterinary Medical Society*.

[13] Gozieva M. (2019). Using modern information technologies in the teaching English language. *Scientific Bulletin of Namangan State University*.

[14] Gu W. X. (2018). Application of learning by design into the cultivation of multiliteracies: a case study of college English teaching practice at Soochow University. *Language & Semiotic Studies*.

[15] Zou D. (2017). Research on college English teaching model based on multimedia and network. *DEStech Transactions on Social Science Education and Human Science*.

[16] Gooch R., Saito K., Lyster R. (2016). Effects of recasts and prompts on L2 pronunciation development: teaching English/ɹ/to Korean adult EFL learners. *System*.

[17] Al-Qallaf C. L., Al-Mutairi A. S. R. (2016). Digital literacy and digital content supports learning. *The Electronic Library*.

[18] Alhassan A. (2017). Teaching English as an international/lingua franca or mainstream standard language? Unheard voices from the classroom. *Arab World English Journal*.

[19] Polat M. (2017). Teachers’ attitudes towards teaching English grammar: a scale development study. *International Journal of Instruction*.

[20] Aljohani O. (2015). Does teaching English in Saudi primary schools affect students’ academic achievement in Arabic subjects?. *Advances in Language and Literary Studies*.

[21] Yang S., Deng B., Wang J. (2020). Scalable digital neuromorphic architecture for large-scale biophysically meaningful neural network with multi-compartment neurons. *IEEE Transactions on Neural Networks and Learning Systems*.

[22] Cai Z., Zheng X. (2020). A private and efficient mechanism for data uploading in smart cyber-physical systems. *IEEE Transactions on Network Science and Engineering (TNSE)*.

[23] Cai Z., Xiong Z., Xu H., Wang P., Li W., Pan Y. (2021). Generative adversarial networks: a survey towards private and secure applications. *Computer Science*.

[24] Liu Y., Ren L. (2022). The influence of artificial intelligence technology on teaching under the threshold of “Internet+”: based on the application example of an English education platform. *Wireless Communications and Mobile Computing*.

